The article "Post-acute (long) COVID-19 quality of life: validation of the German version of (PAC19QoL) instrument" was retracted in 2023. Reasons: plagiarism; overlap with other authors' work.

# Post-acute (long) COVID-19 quality of life: validation of the German version of (PAC19QoL) instrument

**DOI:** 10.3389/fpubh.2023.1163360

**Published:** 2023-06-30

**Authors:** Srikanth Umakanthan, Mariam Monice, Salona Mehboob, Cheryl Linda Jones, Sam Lawrence

**Affiliations:** ^1^Department of Para-Clinical Sciences, Faculty of Medical Sciences, The University of the West Indies, St. Augustine, Trinidad and Tobago; ^2^Independent Researcher, Berlin, Germany; ^3^COVID-19 Independent Research Study Group, Berlin, Germany

**Keywords:** PAC-19QoL, EQ-5D-5L, validation, long COVID-19, questionnaire

## Abstract

**Purpose:**

The aim of our study was to validate a German translation of the post-acute (long) COVID-19 quality of life (PAC-19QoL) instrument among German patients with long COVID-19 syndrome.

**Patients and methods:**

The PAC-19QoL instrument was translated into the German language and administrated to patients with long COVID-19 syndrome. Cronbach's alpha coefficient was used to analyze the internal consistency of the instrument. Construction validity was evaluated by using Pearson's correlation coefficient and Spearman's rank correlation. Scores of patients and controls were compared using the Mann–Whitney *U*-test.

**Results:**

A total of 45 asymptomatic and 41 symptomatic participants were included. In total, 41 patients with long COVID-19 syndrome completed the PAC-19QoL and EQ-5D-5L questionnaires. PAC-19QoL domain scores were significantly different between symptomatic and asymptomatic participants. All items achieved a Cronbach's alpha >0.7. There was a significant correlation between all domains on the test (*p* < 0.001), with the highest correlation between total (*r* = 0.994) and domain 1 (*r* = 0.991). Spearman's rank correlation analysis confirmed that the instrument items correlated with the objective PAC-19QoL examination findings.

**Conclusion:**

The German version of the instrument is valid and reliable and can be a suitable tool for research and daily clinical practice among patients with long COVID-19 syndrome.

## Introduction

As of December 2022, more than 600 million people worldwide have been infected by COVID-19. In Germany, more than 2,650,000 people have been infected (1). Most people with coronavirus (COVID-19) diseases make a full recovery within 12 weeks; however, for some people, symptoms can last longer. This syndrome is called long or post-COVID-19 syndrome. It is a new condition that is still being studied and there are many definitions (2, 3).

According to the World Health Organization (WHO), the post-/long COVID-19 condition occurs in individuals with a history of probable or confirmed SARS-CoV-2 infection, usually 3 months from the onset of COVID-19 with symptoms that last for at least 2 months and cannot be explained by an alternative diagnosis. The most common symptoms are fatigue, shortness of breath, cognitive dysfunction, muscle aches, loss of smell, problems with concentration and memory (brain fog), insomnia, heart palpitations, and others, which generally have an impact on everyday functioning. Symptoms may be a new onset, following initial recovery from an acute COVID-19 episode or persist from the initial illness. Symptoms may also fluctuate or relapse over time (2, 4, 5).

Immune-inflammatory pathways substantially predict the physio-affective phenome in acute and long COVID-19 (6, 7). The lowered peripheral blood oxygen saturation (SpO_2_), increased C-reactive protein (CRP), nitric oxide, increased peak body temperature, lowered antioxidant defenses, such as lowered glutathione peroxidase (Gpx) and zinc levels, and lowered serum calcium reflect the severity of immune-inflammatory response and forecast the physio-affective phenome of prolonged COVID-19 (8, 9). The physio-affective phenome of long COVID-19 predicts the COVID-19 infection–immune-inflammatory pathways during the acute phase of SARS-CoV-2 infection. Furthermore, the nitro-oxidative pathways through the immune inflammation mediate the effects of long COVID-19 as seen in chronic fatigue syndrome/myalgic encephalomyelitis (CFS/ME), bipolar disorder (BD), and major depressive disorder (MDD) (10–12).

Among the specific measures, the five-level EuroQol five-dimensional questionnaire (EQ-5D-5L) is the most recently devised scale. The EQ-5D-5L consists of two parts—the EQ-5D-5L descriptive system (EQ-INDEX) and the EQ visual analog scale (EQ-VAS). The EQ-INDEX comprises five dimensions (mobility, self-care, usual activities, pain/discomfort, and anxiety/depression), and each dimension has five levels: no problems, slight problems, moderate problems, severe problems, and extreme problems. The EQ-VAS is a patient's subjective assessment of generic health ranging from 0 to 100, with higher scores representing better subjective health experience (13). One of the specific disease measures to assess the quality of life of patients with long COVID-19 syndrome is the post-acute (long) COVID-19 quality of life (PAC-19QoL) instrument (14). It is one of the new tools used to assess the quality of life, and therefore, it is not yet widely used or validated in other languages.

The aim of our study was to validate a German translation of the PAC-19QoL instrument among German patients with long COVID-19 syndrome.

## Materials and methods

The original PAC-19QoL instrument was created and validated in English (14). Using a Mann–Whitney *U*-test, statistically significant differences between the mean Likert score for each quality-of-life indicator (variable) were compared between the responses from study participants (both patients and control groups). A *p*-value of <0.05 indicated a statistically significant finding in the presented analyses. All statistical analyses were conducted in R, version 3.6.3. The first step was the author's agreement to translate the instrument into the German language in accordance with standards. Two English expert translators worked independently to produce two German versions of the instrument. After consultation and agreement, one version was selected. The confirmed instrument was interpreted back into the original language to check for any possible content inequality between the original instrument and the final translated version.

The instrument consists of four domains and 19 subdomains:

1. Psychological (mood, isolation, motivation, anxiety, cognition, expression, and mental exertion): items 1–18,
2. Physical (exertion, pain, travel, somnolence, smell/taste, breathlessness, fine motor, and libido): items 19–34,
3. Social (isolation, relationships, and hobbies): items 35–41, and
4. Work (ability to work): items 42–44.

The questionnaire uses a 5-point scoring system. A lower score indicates a better quality of life.

The author of the original instrument was then consulted. After the author's agreement, the final German questionnaire was tested for ambiguous answers among five patients to determine its comprehensibility. The findings from the pilot study were to modify/eliminate certain variables in the questionnaire which did not provide conclusive answers. After this, the final version was created, and it was this version that was used. The next step was the validation of the German version of the instrument.

Participants were identified as asymptomatic when they did not have any persistent symptoms after the outbreak of the COVID-19 disease. Participants were identified as symptomatic/with long COVID-19 syndrome (patients) if they presented symptoms and fulfilled the criteria of long COVID-19 syndrome (The patients who had either a diagnostic or antibody test confirmation for SARS-CoV-2 and were still suffering from post-acute symptoms of COVID-19, were recruited to the study group). All patients seen at the pneumology outpatient clinic were included in the study between September 2022 and December 2022. All participants were aware of the purpose of the study and completed the PAC-19QoL and EQ-5D-5L questionnaires. The authors of this study obtained consent to use the EQ-5D-5L questionnaire. Participants also responded to demographic questions (sex, age, height, weight, the course of COVID-19, persistent symptoms, chronic diseases, abuses, etc.).

PAC-19QoL has been tested for content validity, construct validity, and internal consistency.

### Statistical analysis

The reliability of the instrument was investigated by its internal consistency using Cronbach's alpha. Internal consistency refers to the degree of correlation between the items. A Cronbach's alpha of >0.7 has been recommended as acceptable. The responsiveness of PAC-19QoL and EQ-5D-5L was examined by calculating the standardized response mean and the effect size. To measure the test–retest reliability of the final version, all patients were asked to participate by completing a second instrument (retest) 2 weeks later. The responses of the two completed instruments were then analyzed using Spearman's correlation. Scores of patients and controls were compared using the Mann–Whitney *U*-test. The statistical processing of the results was performed in IBM SPSS Statistics for Windows, version 29.0. We considered a *p*-value of <0.05 to be statistically significant.

The German version of the instrument is shown in Supplementary material.

## Results

A total of 86 participants were enrolled. Of which, 43 participants were symptomatic with long COVID-19 syndrome; however, 41 (93.2%) completed the study and two (6.8%) were excluded (as they failed to follow up during the study period). Men corresponded to 63.4% of the total number. A total of 13 patients (31.7%) were hospitalized due to COVID-19. The average time of hospitalization was 21.62 ± 22.58 days. In total, 29 (70.7%) had a chronic disease (diabetes mellitus, hypertension, stroke, asthma, chronic obstructive pulmonary disease, and high cholesterol). Demographic characteristics of the patients and controls are shown in Table 1.

**Table 1:** Demographic characteristics of the patients and controls (*n* = 86).

**Variables**	**Patients (*n* = 41)**	**Controls (*n* = 45)**	***P*-value**
Male *N* (%)	26 (63.4)	13 (28.8)	0.0013^*^
Age (years; average ± SD)	52.53 ± 12.91	46.28 ± 13.09	0.0287^**^
BMI (average ± SD)	28.24 ± 5.17	25.81 ± 4.94	0.0285^**^
Chronic diseases *N* (%)	29 (70.7)	21 (46.6)	0.0239^*^
Smoking *N* (%)	13 (31.7)	12 (26.6)	0.6539
**Course of COVID-19**			
Hospitalization due to the COVID-19 *N* (%)	13 (31.7)	0 (0)	
Duration of hospitalization (days; average ± SD)	21.62 ± 22.58	0 (0)	
Intensive Care Unit due to the COVID-19 *N* (%)	6 (14.6)	0 (0)	
Duration in intensive care unit (days; average ± SD)	17.33 ± 10.01	0 (0)	
**Long COVID-19 symptoms**			
Duration of long COVID-19 symptoms (days; average ± SD)	560.63 ± 219.38	0 (0)	
Shortness of breath *N* (%)	29 (70.7)	0 (0)	
Fatigue *N* (%)	20 (48.8)	0 (0)	
Muscle ache *N* (%)	11 (26.8)	0 (0)	
Cognitive dysfunction *N* (%)	7 (17.1)	0 (0)	

^*^p < 0.05 (chi-square test); ^**^p < 0.05 (Student's t-test).

N, number; SD, standard deviation.

The mean, standard deviation (SD) of the PAC-19QoL (domains 1–4 and total), and EQ-5D-5L (EQ-INDEX, EQ-VAS) are shown in Table 2.

**Table 2:** Mean scores for PAC-19QoL and EQ-5Q-5L (*n* = 86).

	**Patients (*n* = 41)**	**Controls (*n* = 45)**	
**Instrument scale**	**Mean** ±**SD**	**Mean** ±**SD**	**P value**
Domain 1	44.90 ± 11.6	39.64 ± 7.18	0.0125^*^
Domain 2	45.90 ± 10.46	27.86 ± 6.32	0.0001^**^
Domain 3	16.93 ± 6.55	12.80 ± 3.35	0.0003^**^
Domain 4	8.34 ± 3.47	5.16 ± 1.76	0.0001^**^
Total	115.66 ± 24.93	85.47 ± 13.48	0.0001^**^
EQ INDEX	0.73 ± 0.19	0.87 ± 0.20	0.0013^*^
EQ VAS	63.76 ± 14.05	75.31 ± 17.67	0.0013^*^

^*^p < 0.05, ^**^p < 0.001 (Mann–Whitney U-test).

N, number; SD, standard deviation.

All items achieved a Cronbach's alpha showing acceptable internal consistency. Cronbach's alpha coefficient for variables of the German version of the PAC-19QoL instrument is shown in Table 3.

**Table 3:** Cronbach's alpha coefficient for variables of the German version of the PAC-19QoL instrument (*n* = 41).

**Variable**	**Cronbach's alpha**
Domain 1	0.899
Domain 2	0.864
Domain 3	0.740
Domain 4	0.786
Total score	0.936

There was a significant correlation between all domains on the test (*p* < 0.001), with the highest correlation between total (*r* = 0.994; *p* < 0.001) and domain 1 (*r* = 0.991; *p* < 0.001) (Table 4).

**Table 4:** Reproducibility of PAC-19QoL according to the test–retest (*n* = 41).

**Scores**	PCC^**^	***p*-value**
Domain 1	0.991	<0.001
Domain 2	0.981	<0.001
Domain 3	0.834	<0.001
Domain 4	0.919	<0.001
Total score	0.994	<0.001

^**^PCC Pearson's correlation coefficient.

Spearman's rank correlation analysis confirmed that the instrument items correlated with the objective PAC-19QoL examination findings (Table 5).

**Table 5:** Non-parametric correlations between PAC-19QoL and EQ-5D-5L.

	**Domain 1**	**Domain 2**	**Domain 3**	**Domain 4**	**Total score**
EQ-INDEX	−0.574^**^	−0.523^**^	−0.228	−0.339^*^	−0.565^**^
EQ-VAS	−0.543^**^	−0.577^**^	−0.131	−0.232	−0.559^**^

^*^p < 0.05; ^**^p < 0.01 (Spearman's rank correlation).

The quality of life of long COVID-19 patients in relation to mobility, self-care, and pain/discomfort is shown in Table 6.

**Table 6:** Age group-wise distribution of quality of life in long COVID-19 patients reporting EQ 5D level 1.

	**18–30 years**	**31–40 years**	**41–50 years**	**51–60 years**	**61 and above**
**Mobility**					
1	100	50	0	0	33.3
2	0	50	100	33.3	33.3
3	0	0	0	33.3	0
4	0	0	0	33.3	33.3
5	0	0	0	0	0
**Self-care**					
1	100	50	0	0	0
2	0	50	100	33.3	33.3
3	0	0	0	33.3	33.3
4	0	0	0	33.3	33.3
5	0	0	0	0	0
**Pain/discomfort**					
1	100	50	0	0	0
2	0	50	100	33.3	33.3
3	0	0	0	33.3	33.3
4	0	0	0	33.3	33.3
5	0	0	0	0	0

## Discussion

The quality-of-life assessment (quality-of-life questionnaire) is a very important tool for assessing the course of the disease or its consequences and treatment. An excellent example is the long COVID-19 syndrome; according to many studies, long COVID-19 syndrome results in a poor quality of life in addition to clinical symptoms (15–18). The EQ-5D-3L is found to potentially influence the quality-adjusted life years (QALYs), cost-effectiveness analyses, and results. Even though the EQ-5D-5L questionnaire is the most adopted method, the national sets of assessments are important while considering critical medical conditions and national health states that would create cross-country health disparities and equity issues (16, 17).

The authors of a meta-analysis found that 58% of the long COVID-19 patients had reported poor quality of life. In long COVID-19 patients, the pooled analysis of individual factors in the EQ-5Q-5L questionnaire showed that 41.5% had pain/discomfort, 37.5% had anxiety/depression, followed by 36% had problems with mobility, 28% had problems with usual activities, and only 8% had self-care problems (19). EQ-5D-5L is used to measure the quality of life in patients with long COVID-19 syndrome; it adequately describes the reduction in quality; thus, we chose it as a reference standard for the validation of the PAC-19QoL instrument.

According to authors from France, the mean EQ-VAS was 70.3 ± 21.5, and the mean EQ-5D-5L index was 0.86 ± 0.20. Authors claim that most patients requiring hospitalization for COVID-19 still have persistent symptoms (20). A study conducted by authors from China found that the mean EQ-VAS was 80, and one potential explanation for this phenomenon is that COVID-19 may result in post-traumatic stress disorder (21). For the health-related quality of life, the mean EQ-VAS and EQ-INDEX values in our sample were 63.76 ± 14.05 and 0.73 ± 0.19.

The quality of life for patients with long COVID was higher than that of patients living with type 2 diabetes mellitus (EQ-VAS score was 78.83 ± 15.02) and of patients with multiple sclerosis (65.6 ± 21.5) (22, 23). In our study, the mean EQ-VAS score for patients with long COVID-19 was 72.75 ± 11.05.

Long COVID-19 syndrome is a multisystem disease characterized by a range of symptoms and clinical signs. In this study, the most common symptoms of long COVID syndrome were shortness of breath, fatigue, and muscle pain. The validated instrument contains four domains (psychological, physical, social, and work), which are essential for assessing the quality of life in patients with long COVID-19 syndrome. The questionnaire we used as a reference standard (5Q-5D-5L) contains five domains (mobility, self-care, usual activities, pain/discomfort, and anxiety/depression). Domain 3 (social) of the PAC-19QoL instrument does not correlate with the 5Q-5D-5L questionnaire because this domain concerns social aspects that the reference standard does not. Nevertheless, it is necessary to evaluate the overall quality of life of patients with long COVID-19 syndrome. Finally, the total score correlates with the compared questionnaire; therefore, we evaluated the instrument as suitable.

According to the prospective cohort study from Italy and retrospective study from Iran, the female sex was independently associated with long COVID syndrome. Interestingly, women were characterized by a higher proportion of most physical symptoms and all psychological symptoms than men (24, 25). There were more male participants in our sample; nevertheless, we cannot draw any conclusions based on the small number of patients (but it is sufficient for validation purposes).

Biomarkers strongly predict lower WHO-QoL scores in long COVID-19 (26). The increased PBT and TO2 index (The biomarkers of the acute phase of infection were peak body temperature (PBT) and the lowest SpO2 values. Patients' records are used to acquire PBT) reflect the acute infectious phase of COVID-19 (27, 28). The long COVID-19 is predicted by lowered calcium levels and higher neurotoxins (e.g., OSTOX and NLRP3). Higher levels of peroxides, malondialdehyde, superoxide dismutase, nitric oxide, lower HDL-cholesterol, and paraoxonase 1 (an antioxidant enzyme) are neuro-oxidative toxicity markers which predict lower WHO-QoL scores in patients with BD/MDD (29–31). Kanchanatawan et al. noted that the indices of tryptophan catabolite (TRYCAT) pathway activation with increased production of neurotoxic TRYCATs, such as picolinic acid and xanthurenic acid, was associated with a total WHO-QoL score (32). In a study conducted by Al-Musawi et al., schizophrenia patients showed an inverse relationship between the pathogenic T-helper-17 (Th-17) phenotype and the IL-6/IL-23/Th-17 axis and the WHO-QoL scores (33). In addition, increased levels of tumor necrosis factor (TNF)-α, IL-1β, IL-6, IL-17, IL-21, IL-22, and IL-23 were inversely proportional to the HR-QoL in the schizophrenia patients. Hence, these findings conclude that the neuro-immune and neuro-oxidative stress pathways direct the lower HR-QoL in long COVID-19 patients (34).

In MDD, BD, schizophrenia, and CFS/ME in long COVID-19 are directed by various neuro-oxidative and neuro-immunotoxin pathways. The central circuits that control pain, cognition, memory, sleep, and affection are dysfunctional due to the activation of the neuro-oxidative and neuro-immunotoxin pathways. In MDD, lower calcium, lower insulin resistance, and higher CRP were responsible for pathologic changes in axonal and astroglia cells, causing neuronal injury (35, 36). In patients with unstable angina, activation of immune-inflammatory markers (IL-6 and CRP) is directly related to an increase in insulin resistance and atherogenicity (37). The neurotoxic effects of increased insulin resistance include increased blood–brain barrier permeability, decreased brain-derived neurotrophic factor levels, impaired synaptic plasticity, dendritic spine damage, and decreased hippocampal volume and metabolic activity in the prefrontal cortex (38, 39). Lower serum calcium is not only an indicator of an inflammatory response, but is also associated with psychosomatic symptoms, including muscle spasms and cramps, neuromuscular irritability, paresthesia, circumoral numbness, neurocognitive and memory impairments, fatigue, depression, and anxiety (40–42). Recent meta-analysis findings indicate that low calcium in COVID-19 patients is associated with increased severity, higher mortality, and more complications (43).

Our validation study confirmed very good validity and test–retest reliability of the German version PAC-19QoL. All items achieved a Cronbach's alpha >0.7, which is comparable to the original version.

## Conclusion

We can conclude that the German version of PAC-19QoL is a reliable, consistent, and valid instrument for assessing the quality of life of patients with long COVID-19 syndrome and is a suitable tool for research and daily clinical practice among patients with long COVID-19 syndrome. Due to the large COVID-19-infected population, which has developed long COVID-19 syndrome, we consider the PAC-19QoL instrument to be a unique and specific tool needed for assessing the quality of life among patients with long COVID-19 syndrome. It is necessary to focus on understanding the factors leading to poor quality of life and developing follow-up procedures accordingly. Longer follow-up studies in a larger population are necessary to understand the full spectrum of health and social consequences of COVID-19.

## Data availability statement

The original contributions presented in the study are included in the article/Supplementary material, further inquiries can be directed to the corresponding author/s.

## Ethics statement

The studies involving human participants were reviewed and approved by the Ethics Committee at the University Hospital in Berlin (reference no. EK UNM n. 71/2022). Informed consent was obtained before completing the questionnaire. The patients/participants provided their written informed consent to participate in this study.

## Author contributions

SU: concept, writing original manuscript, and editing. MM, SM, and CJ: data collection, survey tool creation and validation, and statistical analysis. SL: team supervisior. All authors contributed to the article and approved the submitted version.
